# Application of Low-Dose CT and MRI in the Evaluation of Soft Tissue Injury in Tibial Plateau Fractures

**DOI:** 10.1155/2022/7686485

**Published:** 2022-09-16

**Authors:** Yinping Qi, Peipei He, Jianping Zhu, Yanan Wang, Hong Zhao, Junbo Chen

**Affiliations:** Department of Radiology, The Second Hospital of Yinzhou, Ningbo, Zhejiang 315100, China

## Abstract

**Objective:**

To explore the application value of low-dose CT and MRI in the evaluation of soft tissue injury in tibial plateau fractures.

**Methods:**

This study included 89 patients with high suspicion of TPF and KI admitted to our hospital from July 2015 to May 2021. After arthroscopy, 81 patients were diagnosed with FTP combined with KI. The Schatzker classification based on X-ray and CT plain scan combined with three-dimensional reconstruction was recorded, and the soft tissue injury was recorded according to the MRI examination of the affected knee joint.

**Results:**

With the results of pathological examination and arthroscopic surgery as the gold standard, the results of MRI and pathological examination and arthroscopic examination were in good agreement (Kappa = 0.857, 0.844), and CT was moderately in agreement (Kappa = 0.697, 0.694). In KI examination, CT and MRI had no difference in the evaluation of ligament injury and bone injury (*P* > 0.05), but MRI had better diagnostic effect on meniscus injury (*P* < 0.05). Finally, the satisfaction survey showed that patients in the CT group were more satisfied with clinical services (*P* < 0.05).

**Conclusion:**

Both CT and MRI have certain diagnostic value for occult tibial plateau fractures, among which CT examination is more advantageous for trabecular bone fractures, MRI examination is more advantageous for cortical bone fractures, and MRI examination can improve occult tibial plateau fracture inspection accuracy.

## 1. Introduction

Tibial plateau fractures (TPF) refer to a continuous interruption of tibial plateau bone under the action of external forces, mostly commonly seen in motor vehicle accidents or sports injuries, with the symptoms of obvious local pain, swelling, deformity, and dyskinesia [1]. The tibial plateau is an important load structure of the knee joint. Generally, TPF is complicated with knee injuries (KI), which seriously affects patients' daily life. In addition, the rapid development of modern society and various means of transportation all increase the risk of accidents and consequently the incidence of TPF combined with KI [2, 3]. For such patients, timely diagnosis and effective intervention are critical in improving patient prognosis.

X-ray is commonly used in clinical imaging examinations of KI, but still, it has limitations. For example, the diagnosis effect is not comprehensive enough in the face of occult illness or complicated symptoms, and it has certain harm to the human body due to radiation. In addition, the anatomical resolution of X-ray is low due to the overlapping of the patient's bone structures [4]. Especially when the fracture plane is an inclined plane and the articular surface of the tibial plateau collapses, the tissue overlap will lead to the inability to accurately and effectively distinguish the joint injury [5]. Therefore, further arthroscopy is still needed to confirm KI in such patients, which will not only bring secondary trauma to patients with severe bone trauma but also increase the risk of fracture infection and thrombosis [6].

Low-dose CT is an imaging examination clinically advocated at present, which is to diagnose diseases with the minimum scanning range, the lowest dose, and the least X-ray, with less radiation and higher safety compared with traditional X-ray. MRI, another imaging approach, also has a wide range of clinical applications [7]. Using magnetic resonance phenomenon to obtain electromagnetic signals from the human body, it can reconstruct human body information and obtain various physical characteristic parameters of substances and carry out multidirectional imaging. However, we found that there are few clinical reports on the evaluation effects of MRI and low-dose CT on TPF combined with KI [8]. Accordingly, we explored and observed the advantages and disadvantages of the two imaging examinations for the diagnosis of TPF combined with KI, to provide a more efficient and rapid diagnostic method for future clinical treatment.

## 2. Patient Data and Methods

### 2.1. Patient Data

This study enrolled 89 patients with high suspicion of TPF and KI admitted to our hospital from July 2015 to May 2021; after arthroscopy, 81 cases were confirmed to have FTP combined with KI. Inclusion criteria: (1) age 18-80; (2) presence of TPF; (3) MRI and CT examinations were accepted; (4) diagnosis of KI by arthroscopy; (5) surgical treatment in our hospital after admission; (6) time from injury to operation ≤ 1 week; (7) complete medical records. Exclusion criteria: (1) no clear history of trauma; (2) severe diseases of vital organs such as heart, lung, liver, and kidney; (3) coagulation dysfunction; (4) neurological dysfunction or mental disorders; (5) previous TPF history; (6) pregnant and lactating patients.

### 2.2. Inspection Methods

CT examination: a PHILIPS Brilliance 16-slice spiral CT scanner was used to scan patients in the supine position, and the scanning parameters were as follows: voltage 120 kV, current 90 mA, scanning slice thickness 3 mm, matrix 515 × 515, FOV 180 mm × 180 mm, and reconstruction interval 1.0-2.0 mm. After scanning, the original volume data were transferred to the workstation for multiplanar reconstruction (MPR), surface shaded display (SSD), volume rendering (VR), and other processing. MRI: scans were performed using a Kangda 1.5 T MR scanner. Patients were placed in the supine position, and the scanner was used to identify the cross-sectional spin echo (SE) pulse signal with the pulse sequence set as follows: T1WI (TE: 11 ms, TR: 540 ms); T2WI (TE: 80 ms, TR: 3200 ms); layer thickness 8-10 mm, layer spacing 1 mm, field of view 38 cm × 38 cm, and matrix 256 mm × 256 mm.

### 2.3. Evaluation of Image Results

The results of all imaging examinations were double-blindly read by 2 radiologists to evaluate the patient's KI condition. The test result was determined when physicians reached an agreement. And if there was a difference of opinion, a third physician would be consulted. FTP is classified according to the Schatzker classification criteria [9]: type I, split wedge of the lateral tibial plateau; type II, split wedge depression of the lateral tibial plateau; type III, pure depression of the lateral tibial plateau; type IV: split wedge of the medial tibial plateau; type V: bicondylar tibial plateau fracture, where there is continuity between the epiphysis and the diaphysis; type VI: bicondylar fracture with complete dissociation between the epiphysis and the diaphysis.

### 2.4. Outcome Measures

The diagnosis rate of TPF combined with KI by CT and MRI was evaluated, and the evaluation effects of the two inspection methods on the specific injury conditions of KI (including meniscus injury ligament injury and bone injury) were determined. Besides, a satisfaction survey (score range: 0-10) was conducted after surgery, with 10 being very satisfied, 7-9 being satisfied, 4-6 being in need of improvement, and 1-3 being dissatisfied. Overall satisfaction = (very satisfied + satisfied) cases/total cases × 100%.

### 2.5. Statistical Methods

SPSS22.0 software was used for statistical analysis. Quantitative and categorical data were given ‾*χ* (±*s*) and by (%)/[*n* (%)] and compared using the independent samples *t* test and chi-square test, respectively, with *P* < 0.05 indicating statistically significant differences. The Kappa test examined the consistency of MRI and CT with arthroscopic surgery, with a Kappa value > 0.75, 0.4-0.75, and<0.4 indicating good, average, and poor consistency, respectively.

## 3. Results

### 3.1. FTP's Comparison of Inspection Accuracy

Pathological examination confirmed that 84 of 89 patients had FTP; using the results of pathological as the gold standard, the detection rates of KI by CT and MRI were found to be 72 and 82, respectively. MRI showed good consistency with pathological (Kappa = 0.857), while CT showed mediocre consistency (Kappa = 0.697) (Tables 1 and 2).

### 3.2. Types of FTP

Pathological examination results showed that 7 patients were type I, 14 were type II, 8 were type III, 30 were type IV, 16 were type V, and 9 were type VI. CT results showed that 3 patients were type I, 17 were type II, 6 were type III, 23 were type IV, 15 were type V, and 8 were type VI. MRI results showed that 8 patients were type I, 15 were type II, 8 were type III, 28 were type IV, 14 were type V, and 9 were type VI. Compared with pathological examination, both CT and MRI have excellent diagnostic performance for FTP typing (*P* > 0.05) (Tables 3 and 4).

### 3.3. KI's Comparison of Inspection Accuracy

Arthroscopic examination confirmed that 81 of 89 patients had FTP combined with KI; using the results of arthroscopy as the gold standard, the detection rates of KI by CT and MRI were found to be 63, and 77, respectively. MRI showed good consistency with arthroscopy (Kappa = 0.844), while CT showed mediocre consistency (Kappa = 0.694) (Tables 5 and 6).

### 3.4. CT and MRI Diagnosis of Meniscus Injury

Arthroscopy showed meniscus injury in 42 cases, while MRI diagnosis of meniscus injury in 41 cases showed high signal intensity on T2WI with elliptical, spherical, patchy, or linear distribution. CT examination diagnosed 37 cases of meniscus injury, with visible changes in meniscus morphology, loss of smooth edges, and visible bone fragments. After calculation, it was found that MRI had higher sensitivity, specificity, and accuracy in the diagnosis of meniscus injury than CT (*P* < 0.05) (Table 7).

### 3.5. Diagnostic Efficacy of CT and MRI for Ligament Injury

Arthroscopy showed 39 cases of ligament injury, including 17 of anterior cruciate ligament injury (3 of complete tear, 8 of partial tear, and 6 of rubbing); 10 of posterior cruciate ligament injury (2 of complete tear, 6 of partial tear, 2 of rubbing); 6 of medial collateral ligament injury; 4 of lateral collateral ligament injury; 2 of multiple ligamentous mixed injuries. MRI examination diagnosed 43 cases of ligament injury, and the main imaging manifestations were as follows: ligament contusions showed ligament thickening with undulating edges and high signal intensity on T1 and T2; partial tears of the ligament presented with uneven signals of the ligament accompanied by some abnormally high signals, but the ligament continuity was not interrupted; complete ligament tears were characterized by loss of ligament continuity, disappearance of ligament shadow, and irregular abnormally high signal intensity. 40 cases of ligament injury were diagnosed by CT. On CT scans, ligament contusions were manifested as thickened ligament, decreased density, and unclear surrounding adipose space; ligament tears were characterized by ligament contracture and swelling, as well as discontinuity and low density of the ligament. No statistical difference was determined in the sensitivity, specificity, and accuracy of MRI and CT in diagnosing ligament injury after calculation (*P* > 0.05) (Table 8).

### 3.6. Diagnostic Efficacy of CT and MRI for Bone Injury

Arthroscopy confirmed bone injury in 22 cases. 23 cases of bone injury were diagnosed by MRI, and the images showed low and isointensity on T1 while isointensity and high signal on T2. CT examination diagnosed bone injury in 25 cases, with obvious fracture lines found on images. After calculation, it can be seen that the sensitivity, specificity, and accuracy of MRI and CT in the diagnosis of ligament injury were not statistically different (*P* > 0.05) (Table 9).

## 4. Discussion

As we all know, the tibia, the most common fracture site in the human body, is also a key site that affects normal human walking and activities. The knee joint connected with the tibial plateau is one of the most important joint activity centers in the human body and also the most complex and frequently used flexion joint [10]. Although the occurrence of tibial fracture or KI can be diagnosed quickly and accurately by CT, MRI, X-ray, and other imaging methods at present, there is still a lack of reliable studies to provide reference for patients with TPF combined with KI. Therefore, a more secure and reliable means to evaluate TPF patients with KI is of great significance to ensure the rehabilitation and safety of patients.

MRI and CT, as the most classic and common imaging modalities, have a relatively stable evaluation effect for KI [11]. But their employment in TPF patients with KI is rarely reported, which warrants further investigation regarding their evaluation effects in such a patient population. Therefore, by comparing the merits and demerits of MRI and CT in evaluating TPF combined with KI, this study has profound reference significance for the future clinical diagnosis and treatment of such patients. In addition, the low-dose CT used in this study has higher safety for patients and can effectively reduce radiation injury during CT examination, which also enjoys wider clinical application potential.

Herein, we first compared the diagnostic accuracy of CT and MRI, and the results showed that MRI had a more ideal detection rate for TPF complicated with KI. At present, CT examination can only diagnose joint dislocation and fracture, but it is difficult to accurately diagnose cartilage fracture and meniscus injury [12]. MRI, on the other hand, has high resolution for blood vessels, soft tissue synovium, nerves, tendons, muscles, ligaments, and hyaline cartilage, which makes it feasible for clinical examination of hyaline cartilage degeneration and ischemic necrosis, cruciate ligament injury, knee meniscus, as well as osteomyelitis and neurologic complications of rheumatoid diseases [13, 14]. As we all know, the principle of MRI inspection is to place the human body in a special magnetic field, so that the radio frequency pulse reacts with the hydrogen nuclei in the human body to generate hydrogen nucleus resonance. After the radio frequency pulse stops, the hydrogen nuclei can emit radio signals according to their specific frequencies and form images through computer processing [15]. MRI, as a three-dimensional cross-sectional imaging, can obtain multidirectional examination images of patients without reconstruction, whereas the examination time and cost are high, and it is not suitable for patients with metal implants. Therefore, in the examination of fracture patients complicated with KI, MRI cannot be performed if the patient has undergone metal internal fixation. CT examination has no above limitations with higher clinical applicability, but its imaging results for body tissues are not as clear as MRI, which is also one of the main shortcomings [16]. In this paper, we found that MRI has excellent accuracy in diagnosing meniscus injury. This is due to the increase of hydrogen protons in fibrocartilage and the infiltration of synovial fluid during meniscus damage, which turns the original low signal into high signal [17], so MRI can accurately identify meniscus injury, while CT relies on observation of meniscus morphological changes and edge smoothness for judgment [18], and it may not be able to present the full view of the meniscus from the same level when complicated with TPF, which may easily lead to missed diagnosis and misdiagnosis. Subsequently, in the assessment of ligament injury, we found no significant difference in the diagnostic performance between MRI and CT. Knee ligament injury often causes bleeding, edema, etc. MRI findings of the injured site may show obvious abnormal high signal intensity, as well as the loss of signal continuity of the ligament, showing irregular waves [19]. The imaging effect of CT for ligament injury is not as significant as that of MRI. However, with the rapid development of CT technology and the application of three-dimensional reconstruction technology in recent years, the definition of CT images has been improved, which can better present the structure and injury of the cruciate ligament and improve the accuracy of CT diagnosis of ligament injury through multilevel observation of bone and ligament [20]. In addition, in the evaluation of bone injury, the diagnostic performance of the two examination methods also shows obvious differences. MRI can effectively display bone injury and has different signal sensitivity to knee joint soft tissue of patients, with the characteristics of broad field of vision and multidirectional imaging, allowing for higher resolution and effective judgment of bone injury severity [21]. And although CT has a low resolution for soft tissue examination, it has an ideal evaluation effect for bone tissue [22]. In previous studies, we also found consistent performance of MRI and CT in evaluating bone injury in KI, which corroborated our results. Finally, the satisfaction survey results showed that patients in the CT group had a higher evaluation of clinical service quality, which we believe is also related to the longer examination time and higher cost of MRI. However, due to the reduction of voltage, current, and exposure time during CT examination, low-dose CT images are often considered to be not clear enough to meet the needs of clinical evaluation, while this study showed that low-dose CT also had an excellent effect in FTP combined with KI, which is speculated to be due to the large difference in texture and density between knee bone and joint tissues and surrounding tissues. But in the examination of other human tissues, the quality of the image results of low-dose CT should be taken into consideration although it can effectively reduce radiation damage.

## 5. Conclusion

Both low-dose CT and MRI have excellent results in the evaluation of TPF combined with KI, of which the latter is more effective in diagnosing meniscus injury but with more complicated procedures and higher cost. In the actual clinical diagnosis, clinicians should choose the best diagnosis techniques for patients based on their specific conditions and family economic status. It is suggested that when evaluating patients with FTP complicated with KI, low-dose CT should be used for preliminary screening to identify the type of KI while ensuring less radiation damage, and MRI can be further applied to improve the diagnosis when low-dose CT cannot complete the evaluation.

## Figures and Tables

**Table 1:** CT detection of FTP.

Arthroscopy	CT		Total	Kappa	*P*
	(+)	(-)			
(+)	69	15	84	0.697	0.034
(-)	3	2	5		
Total	72	17	89		

**Table 2:** MRI detection of FTP.

Arthroscopy	CT		Total	Kappa	*P*
	(+)	(-)			
(+)	82	2	84	0.857	0.009
(-)	0	5	5		
Total	82	7	89		

**Table 3:** CT results of FTP typing.

	Total	Type I	Type II	Type III	Type IV	Type V	Type VI
CT	72	3	17	6	23	15	8
Pathological examination	84	7	14	8	30	16	9
*χ* ^2^		1.122	1.174	0.067	0.246	0.078	0.006
*P*		0.290	0.279	0.795	0.620	0.781	0.937

**Table 4:** MRI results of FTP typing.

	Total	Type I	Type II	Type III	Type IV	Type V	Type VI
MRI	82	8	15	8	28	14	9
Pathological examination	84	7	14	8	30	16	9
*χ* ^2^		0.102	0.076	0.003	0.004	0.109	0.003
*P*		0.749	0.783	0.960	0.832	0.741	0.957

**Table 5:** CT detection of KI.

Arthroscopy	CT		Total	Kappa	*P*
	(+)	(-)			
(+)	57	24	81	0.694	0.039
(-)	6	2	8		
Total	63	26	89		

**Table 6:** MRI detection of KI.

Arthroscopy	MRI		Total	Kappa	*P*
	(+)	(-)			
(+)	75	6	81	0.844	0.016
(-)	2	6	8		
Total	77	12	89		

**Table 7:** Diagnostic efficacy of CT and MRI for meniscus injury.

	Sensitivity	Specificity	Accuracy
CT	72.97%	65.91%	69.14%
MRI	90.24%	87.50%	88.89%
*χ* ^2^	3.939	5.384	56.760
*P*	0.047	0.020	<0.001

**Table 8:** Diagnostic efficacy of CT and MRI for ligament injury.

	Sensitivity	Specificity	Accuracy
CT	87.50%	90.24%	88.89%
MRI	88.37%	97.37%	92.59%
*χ* ^2^	0.015	1.689	0.661
*P*	0.903	0.194	0.416

**Table 9:** Diagnostic efficacy of CT and MRI for bone injury.

	Sensitivity	Specificity	Accuracy
CT	80.00%	91.30%	91.30%
MRI	95.65%	98.28%	96.30%
*χ* ^2^	2.683	2.108	1.705
*P*	0.101	0.147	0.192

## Data Availability

The data used to support the findings of this study are available from the corresponding author upon request.
